# Study on the Influence of Urban Built Environment Factors on the Social Behavior of ASD Children

**DOI:** 10.1155/2022/8963416

**Published:** 2022-10-12

**Authors:** Shengzhen Wu, Pohsun Wang, Lihao Yao

**Affiliations:** ^1^Faculty of Innovation and Design, City University of Macau, Macau 999078, China; ^2^State Key Laboratory of Subtropical Building Science, South China University of Technology, Guangzhou, 510641 Guangdong, China; ^3^College of Coastal Agricultural Sciences, Guangdong Ocean University, Zhanjiang, 524000 Guangdong, China; ^4^School of Architecture and Urban Planning, Zhuhai College of Science and Technology, Zhuhai, 519041 Guangdong, China

## Abstract

The use of urban space by vulnerable groups, especially ASD children with social anxiety, is an important part of building sustainable urban development. In this study, we focus on the play behavior of ASD children from the perspective of urban planning; then, we discussed how the urban built environmental factors affect the social behavior of ASD children. In this paper, 220 parents of ASD children were given questionnaires and 197 valid questionnaires were obtained after removing invalid ones. Stepwise regression was adopted to further accurately analyze the influence of each factor index in the built environment on children's social behavior. The results showed that multiple urban built environment factors had significant influence on the social behaviors (observation, participation, retreat, and concealment) of children with autism at three stages: before departure, during journey, and arrived at destination. The purpose of study is to fully consider the use of urban space by ASD children when urban researchers or urban planners construct sustainable urban forms, formulate urban design guidelines, and implement old city renewal strategies.

## 1. Introduction

Autistic spectrum disorder (ASD) is listed by the WHO as the first mental disease that seriously affects children's health in global public health problems. Among them, social disorder is the core problem of children who suffer from ASD (Hereinafter referred to as ASD children), which has a far-reaching impact on children's social activities. If it is not treated in time, it will have a great impact on children's living ability and social function [1]. Therefore, this study discusses how the built environmental factors affect the social behavior of ASD children, so as to provide a new vision for urban planning and building a child-friendly city. At the same time, we also pay attention to vulnerable groups, take ASD children as a medium, and then explore the sustainable development of the city in view of social equity.

The Diagnostic and Statistical Manual of Mental Disorders (DSM-V, American) believes that ASD children have social anxiety in specific fear situations [2]. According to the Chinese classification of mental disorders (CCMD-3, China), they will try their best to avoid what they fear or endure it with fear [3]. There are significant characteristics of social anxiety in ASD children: one is the persistent anxiety in social situations; the second is the inability to control this social anxiety. Play behavior is considered as a major behavior of children, which can promote social interaction between children and others [4]. Studies have shown that if ASD children play pretend games, their social ability will be improved [5]. Moreover, gaming has a positive impact on children's mental health, thus alleviating social anxiety and improving the possibility of social behaviors [6]. Therefore, we have reason to believe that the social behavior of ASD children is closely related to the play behavior and the play behavior can represent the social behavior. Children's play behavior is generally divided into the following steps [7]:

1. Observation. Children observe the behavior of other children to further judge whether they have the willingness to participate in the activities that other children are engaged in
2. Participation. After preliminary observation and judgment, children will try their best to join in but it may not be accepted. If rejected, children may still take some behaviors to join in, such as quietly blending in and sharing items
3. Retreat. When children lose interest or confidence in activities, they have withdrawal behavior, which manifests as withdrawing from social situations
4. Concealment. When children are tired or afraid, they will look for quiet rest space where they can be alone. Enclosed space with strong sense of privacy is easy to bring children a sense of security

Fyhri et al. studied the independent mobility of children to schools, friends, and places of leisure activities through the 2005 Norwegian National Tourism Survey and telephone interviews on children's living physical environment and activities. A structural equation model was used to investigate the impact of a range of background variables on the choice of schooling or leisure activity patterns among Norwegian children. The study found that the distance to school and the age of children were the most influential variables on the independent mobility of children, and there were significant seasonal differences in travel modes, and the overall travel level was low in winter. Objective descriptions (subjective assessments) of the traffic environment indirectly explain independent mobility through parents' experience of how safe roads are to go to school. Jiayao et al. investigated how a built environment affects children's independent walking to and from school by means of questionnaire survey and analyzed students from three primary schools in Wenshan, Zhongnan, Jingmei, and Xinhua in Taipei. The analysis results showed that higher shade density and higher sidewalk coverage encouraged children to walk to and from school independently, while a larger block size and increased number of intersections discouraged children from walking to and from school independently. In addition, while high building density, high vehicle density, and diverse commuting options encourage children to walk home from school, a bus or medium passenger transport, block size, and road width discourage children from walking. The study also proposes three strategies to reshape Taipei's built environment: compact structures, pedestrian-friendly designs, and frequent bus services. This study explores the interaction between children and their peers. The target population is ASD children whose behavior is highly dependent on parents and whose social behavior is in the basic stage. Through the questionnaire survey of parents, more real feedback can be obtained. According to previous interviews, ASD children often travel mainly by walking accompanied by their parents. Therefore, this study is aimed at exploring the influence of built environment on children's social behavior by representing social behavior through game behavior after a random trip. It should be noted that open space and semiopen space are the research scope of this study is and do not pay attention to an indoor environment.

According to the travel process, the built environment factors are matched (Table 1):

1. Before departure (building density). Overcrowded housing conditions have a negative impact on the healthy development of children [8]
2. During journey (traffic environment, road environment). Children's physical activities and outdoor games are positively correlated with the walking path, bicycle path, road connectivity, park accessibility, recreational facilities, destinations, and public transportation in the built environment; it is negatively correlated with high traffic exposure and crime [9, 10]
3. Arrived at destination (population density, environmental safety, environmental quality, and land use). Children's play behavior is related to parents' cognition of the built environment. Facilities (parks and play spaces, street lighting, sidewalks and roads, public transportation, shops, and basic services), safety and cleanliness of destinations, population density, and surrounding greening degree all have an impact on children's play behaviors [11, 12]

## 2. Method

The participants in this study were parents of ASD children in special education schools in Fujian province, China. At the beginning of the study, we contacted the principal through the Internet, introduced the intention and method of the study through video clips, and invited the principal to spread the questionnaire to the parents of the children and through the “snowball” approach to more principals, to obtain their assistance.

This study focuses on three core issues: how the built environment before departure affects the social behavior of ASD, how the built environment during journey affects the social behavior of ASD, and how the built environment arrived at destination affects the social behavior of ASD. The dependent variable is the social behavior (observation, participation, retreat, and concealment) of ASD children, and the independent variable is the built environmental factor during the travel process (before departure, during journey, and arrived at destination).

In this study, an online questionnaire was distributed to parents of ASD children. Parents will be asked to take their children to destinations that are 5–10 minutes' walk away from where they live, such as parks. The first part of the questionnaire describes children's gender, age, family background, etc. The second part is based on parents' objective cognition of built environment and children's actual play behavior. The second part was based on the travel process (before departure–during journey–arrived at destination), and the built environment factors (building density, traffic, road environment, population density, environmental safety, environmental quality, land use, and children's games behavior) on children's journey will be completely divides to the above three processes. The questions were positively described (e.g., is there a good sidewalk facility between your residence and destination?); the answers are as follows: “strongly agree,” “agree,” “not necessarily,” “disagree,” and “strongly disagree,” which are marked as 5, 4, 3, 2, and 1, respectively.

This research method is a combination of quantitative and qualitative research methods. The questionnaire is a subjective survey, which is used as the dependent variable after reliability and validity analysis. The objective built environment is the objective data, which is used as the independent variable. Multiple regression was used to explore the causal relationship between dependent variables and independent variables.

Open space and semiopen space are the research scope of this study, which expands the comprehensiveness of the research. In addition, autistic children and the research on vulnerable groups are the research object, which also enriches the theoretical knowledge of the built environment.

## 3. Result

Parents of 220 ASD children were invited to participate, but only 197 parents submitted valid questionnaires. There was only one difference in gender among the subjects. The age distribution is mainly concentrated in 6–9 (42 children aged 3–6 and 41 children aged 9–12). Of all the respondents, 67% have registered permanent residence and only 7.5% are single-parent families. 31% had parents and children living together, and 69% had parents, children, and grandparents living together. Most of the total household income was 10000–20000 RMB per month, accounting for 61.5% of the total. The educational background of the main guardians in their families is high school, accounting for 48.5%, followed by bachelor's degree or above, accounting for 38%. About 49.5% of families have two children, followed by the only child, accounting for 41%. 67% of the children in other families are healthy, 20% are subhealthy, and 13% have physical or mental defects.

As there are variables involved in the distance and destination, some coefficients are not significant in the regression analysis, which does not contribute to the goodness of *R* squared. Therefore, stepwise regression is adopted in the regression part to further accurately analyze the influence of each indicator in the built environment on children's outdoor activities and games (which is described as follows as social behavior, and social behavior includes observation, participation, retreat, and concealment).

### 3.1. How the Built Environment before Departure Affects the Social Behavior of ASD

At the significance level of 0.01, residential building density has a positive influence on the four behaviors of children (Table 2). This happens to coincide with the positive correlation between children's activities and residential density found in previous literature studies [13]. Residential building density and residential greening degree have a positive impact on children's retreat and conceal behavior. Higher building density means more complex spatial relations and higher population density, which are positively correlated with ASD children's social retreat behavior [14]. Exposure to green space can effectively promote mental health [15] and increase the possibility of children's social behaviors (Table 2).

### 3.2. How the Built Environment during the Journey Affects the Social Behavior of ASD

At the significance level of 0.01, intersection environment and complete sidewalk facilities have a positive impact on children's observation behavior (Table 3). At the significance level of 0.05, children's observation behavior was positively affected by traffic light waiting affecting the observation behavior of arriving at the destination.

When the significance level was 0.01, destination accessibility, sidewalk greening, and vehicles yield to pedestrians had a positive impact on children's participation behavior. The perception of road environmental safety can improve children's enthusiasm in activities [16]. The proportion of green plants, pedestrian-friendly traffic environment, and accessibility of leisure areas can support children's active lifestyle and independent mobility [17]. However, when the significance level is 0.05, isolation facilities for people and vehicles and roadside parking have a positive impact on children's participation behavior [18, 19].

When the significance level was 0.01, sidewalk facilities, roadside parking, and road connectivity had a positive impact on children's withdrawal behavior. By reducing the number of roadside parking spaces, the proportion of children's activities can be effectively increased [20]. At the significance level of 0.05, the intersection environment and sidewalk greening had positive effects on children's retreat behavior. The number of intersections and road connectivity have a negative impact on children's outdoor activities [21].

When the significance level was 0.01, the accessibility of destination, sidewalk greening, and vehicle comity had a positive impact on children's concealed behavior. Children with autism experience the stress-relieving benefits of nature more than typically developing children [22]. At the significance level of 0.05, isolation facilities for people and vehicles and roadside parking had a positive impact on children's participation behavior. Isolation facilities for people and vehicles mean safety and have a positive impact on children's activity behaviors [19].

When the significance level is 0.01, the number of activity facilities, complete leisure facilities, quality of leisure facilities, and the number of activity venues have a significant positive impact on children's participation behavior. Improving the quantity and quality of community and park infrastructure (such as recreational facilities, rest seats, and dustbins) may have a positive impact on the activities of children and adults [23, 24]. Parents' awareness of the environment will affect children's activity level [25]. In addition, the preliminary field observation also found that parents would give priority to places with more age-appropriate facilities when choosing destinations and these places are often visited, which also well explains the possibility that children can get more participation in familiar places (Table 4).

When the significance level was 0.01, the number of children, noise interference, the number of activity facilities, and the quality of leisure facilities had a significant positive impact on children's retreat behavior. ASD children are more sensitive to sound than ordinary people [26], and excessive noise will lead to high response of their sympathetic nervous system, which is related to problem behavior and pain [27]. However, when the significance level was 0.05, only the destination monitoring function had a significant positive effect on children's retreat behavior. Parental monitoring has a strong negative impact on children's activities, while the presence of other active children has a strong positive correlation with sports activities in parks [28]. However, in this study, the monitoring function comes not only from parents but also from some electronic monitoring facilities and the crowd. In addition, in the preliminary observation, it is found that parents will consciously guide children in their gaming behaviors, so children's retreat behavior at the destination will be affected by both the population density and the monitoring function.

At the significance level of 0.01, a clean environment, the number of activity venues, and lighting equipment have a significant positive impact on children's concealment behavior. ASD children have difficulty initiating and responding to social interactions with others, maintaining eye contact, sharing objects and activities, and responding to others' feelings [29]. In one of the early observations, a child was socially interrupted by inappropriate behavior and then went straight to another play space, avoiding the previous social situation. It shows that with more playgrounds in the destination, the ASD children may be able to hide themselves by leaving the current playgrounds and entering new ones. Children's vitality is positively correlated with the strength of lighting equipment [30]. Places with sufficient light often improve children's sense of security, which also explains the behavior of ASD children who tend to hide themselves in their parents' arms or some private space after being frustrated in games. However, when the significance level is 0.05, complete service facilities and monitoring function have a significant positive impact on children's concealment behavior. One study confirmed that children with ASD spend more time on aimless activities, interact less with others, and maintain a greater physical distance from their peers than their typically developing peers [31]. The more services a destination has, the more people it is likely to attract to use it, which is one of the reasons why ASD children have difficulty maintaining normal social behavior.

## 4. Discussion

This study focuses on the built environment for autistic children's activities, including open space and semiopen space and indoor environment (such as house, bedroom, kindergarten, social welfare institution, hospital, and rehabilitation center). Therefore, it can be further studied as another study question in future research. At the same time, due to the difficulty in finding samples, this study was only conducted on autistic children in one city in China, which limited the external validity of the research conclusions. If conditions permit in the future, studies on autistic children in different types of cities can be conducted and the comparative study concludes that there are differences.

## 5. Conclusion

In the context of the global construction of a “child-friendly city” and “healthy city,” this study focuses on the vulnerable group of children, ASD children. The improvement of the built environment can improve the social behavior of ASD children and alleviate their social anxiety. The empirical analysis draws the following conclusions and suggestions:

For the residential environment, appropriate control of building density in residential areas can increase the social behavior of ASD children upon arrival at their destination. Increasing the proportion of residential greening can not only promote the physical and mental health of ASD children but also play a significant role in promoting their social behavior in the destination. Therefore, the greening area should be increased in urban planning and design.

For the environment during journey, increasing sidewalk facilities at intersections and reducing waiting time at traffic lights, strengthening traffic control, enforcing speed limits by sections, and increasing roadside no-stop zones can promote pedestrian-oriented travel. At the same time, the establishment of green space with moderate distance, the increase of separation facilities between people and vehicles, and the reasonable division of no parking area for vehicles can also improve the possibility of social interaction of ASD children.

For the destination environment, keeping the environment clean and odor free, setting up a variety of activity venues with different functions, limiting the theme of the venue (such as a special children's park), and increasing the number of activity facilities can improve the observation behavior of ASD children. Increasing the completeness of leisure facilities (such as adding pavilions, landscape corridors, rest seats, and other facilities for people to rest) and improving the quality of leisure facilities can promote the participation behavior of ASD children. Controlling the crowd density of the destination, reducing noise interference, and increasing monitoring functions (such as setting up enough monitoring equipment and increasing patrol security personnel) can reduce the withdrawal behavior of ASD children and maintain the social process. Keeping the destination environment clean and tidy (such as without sundry and garbage being discarded), increasing the lighting equipment, and completeness of service facilities (such as toilet, canteens, and other infrastructure services) to the concealment behavior of ASD children have a positive role in promoting, can protect them after social rejection, and get enough security requirements.

## Figures and Tables

**Table 1:** Description of built environment factors based on the travel process.

Travel process	Built environment elements	Element details
Before departure	Building density	Residential building density, residential greening degree
During journey	Traffic environment	Accessibility of destination, complete sidewalk facilities, traffic light waiting time, intersection environment
	Road environment	Sidewalk greening, sidewalk shading, isolation facilities for people and vehicles, roadside parking, vehicle occupancy on sidewalks, road connectivity, number of vehicles, vehicle speed, vehicles yield to pedestrians
Arrived at destination	Population density	Crowd density, number of children
	Environmental safety	Greening degree, noise interference, no peculiar smell, clean environment, building form
	Environmental quality	Safety, lighting equipment, monitoring function, private space, convenient transportation, safe intersection
	Land use	Complete service facilities, type of activity facilities, number of activity facilities, quality of active facilities, complete leisure facilities, number of leisure facilities, quality of leisure facilities, complete activity venues, number of activity venues, quality of activity venues

**Table 2:** Linear regression analysis of the before departure built environment on social behavior of ASD children.

Variables	Observation	Participation	Retreat	Concealment
Residential building density	0.596^∗∗∗^	0.411^∗∗∗^	0.408^∗∗∗^	0.486^∗∗∗^
Residential greening degree	0.259^∗∗∗^	0.467^∗∗∗^	0.284^∗∗∗^	0.354^∗∗∗^
Constant	0.662^∗∗∗^	0.477^∗∗^	1.369^∗∗∗^	0.622^∗∗^
*F*-Statistic	154.28^∗∗∗^	129.13^∗∗∗^	100.92^∗∗∗^	101.49^∗∗∗^
Observations	200	200	200	200
*R* squared	0.610	0.567	0.506	0.507
Adj *R* squared	0.606	0.563	0.501	0.502

Robust *t*-statistics in parentheses; ^∗∗∗^*p* < 0.01, ^∗∗^*p* < 0.05, and ^∗^*p* < 0.1.

**Table 3:** Linear regression analysis of the during journey built environment on social behavior of ASD children.

Variables	Observation	Participation	Retreat	Concealment
Accessibility of destination		0.177^∗∗∗^		0.193^∗∗∗^
Complete sidewalk facilities	0.192^∗∗∗^		0.204^∗∗∗^	
Traffic light waiting time	0.194^∗∗^			
Intersection environment	0.234^∗∗∗^		0.174^∗∗^	
Sidewalk greening		0.265^∗∗∗^	0.150^∗∗^	0.204^∗∗∗^
Isolation facilities for people and vehicles		0.161^∗∗^		0.148^∗∗^
Roadside parking		0.133^∗∗^	0.224^∗∗∗^	0.127^∗∗^
Vehicle occupancy on sidewalks	0.183^∗∗^			
Road connectivity			0.209^∗∗∗^	
Vehicle speed	0.167^∗∗^			
Vehicles yield to pedestrians		0.301^∗∗∗^		0.185^∗∗∗^
Constant	0.025	−0.173	0.132	0.608^∗∗^
*F*-Statistic	63.19^∗∗∗^	77.44^∗∗∗^	71.23^∗∗∗^	51.98^∗∗∗^
Observations	200	200	200	200
*R* squared	0.620	0.666	0.647	0.573
Adj *R* squared	0.609	0.657	0.638	0.562

Robust *t*-statistics in parentheses; ^∗∗∗^*p* < 0.01, ^∗∗^*p* < 0.05, and ^∗^*p* < 0.1.

**Table 4:** Linear regression analysis of the arrived at destination built environment on social behavior of ASD children.

Variables	Observation	Participation	Retreat	Concealment
Number of children			0.253^∗∗∗^	
Noise interference			0.256^∗∗∗^	
No peculiar smell	0.206^∗∗∗^			
Clean environment				0.196^∗∗∗^
Building form	0.214^∗∗∗^			
Complete service facilities				0.156^∗∗^
Number of activity facilities	0.175^∗∗^	0.277^∗∗∗^	0.228^∗∗∗^	
Complete leisure facilities		0.310^∗∗∗^		
Quality of leisure facilities		0.244^∗∗∗^	0.193^∗∗∗^	
Complete activity venues	0.179^∗∗∗^			
Number of activity venues		0.217^∗∗∗^		0.207^∗∗∗^
Safety	0.258^∗∗∗^			
Lighting equipment				0.198^∗∗∗^
Monitoring function			0.180^∗∗^	0.124^∗∗^
Constant	−0.220	−0.229	0.641^∗∗∗^	0.524^∗∗^
*F*-Statistic	67.81^∗∗∗^	89.12^∗∗∗^	69.35^∗∗∗^	68.33^∗∗∗^
Observations	200	200	200	200
*R* squared	0.636	0.646	0.641	0.637
Adj *R* squared	0.627	0.639	0.632	0.629

Robust *t*-statistics in parentheses; ^∗∗∗^*p* < 0.01, ^∗∗^*p* < 0.05, and ^∗^*p* < 0.1.

## Data Availability

The data used to support the findings of this study may be released upon application to the ethics committee of the school of architecture and urban planning, Zhuhai College of Science and Technology, who can be contacted at the following email address: arczcst@163.com.

## Appendix

### A.1. Description of the Research Process

The sources of the research object are Li Yanyu by Jinjiang city special education school principal help, further through the school teachers and the foundation of Xiamen New Hin Lee secretary general, Zhangzhou Angle beauty Huang Jiehong town special education school principal, Miss Huang Xiamen autism rehabilitation institutions, Xiamen Tongan district special education school principal, Lin Wang Jinjiang psychiatric hospital doctors, and others.

Collect individual data by using the “Wenjuan star online questionnaire collection tool.” First, upload the questionnaire questions and answer options through the online platform of Wenjuan star and distribute the questionnaire links generated by the platform to parents and friends. The questionnaire was officially released and launched on October 1, 2020, with a total of 270 copies pushed. At the same time, on December 24, 2020, 200 valid questionnaires were collected after eliminating invalid questionnaires (for example, the answer time was decisive, the answers were the same, and they were the first option of each question), which were used as basic data to analyze “the influence of the urban built environment based on parents' subjective cognition on the social behavior of children with autism.”

## Additional Points

*Institutional Review Board Statement.* Ethical review and approval were waived for this study due to expediting procedure under the COVID-19 pandemic. However, before the beginning of this study, the purpose of this study and matters needing attention have been explained to the participants through video explanation.
